# Self-organization of intracellular gradients during mitosis

**DOI:** 10.1186/1747-1028-5-5

**Published:** 2010-01-29

**Authors:** Brian G Fuller

**Affiliations:** 1 Department of Biochemistry and Molecular Genetics, University of Virginia, School of Medicine, Charlottesville, Virginia, 22908, USA

## Abstract

Gradients are used in a number of biological systems to transmit spatial information over a range of distances. The best studied are morphogen gradients where information is transmitted over many cell lengths. Smaller mitotic gradients reflect the need to organize several distinct events along the length of the mitotic spindle. The intracellular gradients that characterize mitosis are emerging as important regulatory paradigms. Intracellular gradients utilize intrinsic auto-regulatory feedback loops and diffusion to establish stable regions of activity within the mitotic cytosol. We review three recently described intracellular mitotic gradients. The Ran GTP gradient with its elaborate cascade of nuclear transport receptors and cargoes is the best characterized, yet the dynamics underlying the robust gradient of Ran-GTP have received little attention. Gradients of phosphorylation have been observed on Aurora B kinase substrates both before and after anaphase onset. In both instances the phosphorylation gradient appears to result from a soluble gradient of Aurora B kinase activity. Regulatory properties that support gradient formation are highlighted. Intracellular activity gradients that regulate localized mitotic events bare several hallmarks of self-organizing biologic systems that designate spatial information during pattern formation. Intracellular pattern formation represents a new paradigm in mitotic regulation.

## Introduction

Spatial regulation during mitosis makes possible the equitable distribution of genetic material among daughter cells. Recent observations suggest that cells utilize intracellular gradients as the basis for the spatial regulation of mitotic events [1-7]. In the animal cell lacking existing basal or apical polarity, the metaphase plate and equatorial division plane have no known pre-determined location. Rather, mitotic chromatin provides a 'signal' [8] that focuses the intrinsic self-organizing power of microtubules, motor proteins and microtubule regulators to produce a functional spindle capable of establishing bipolar kinetochore attachments, congressing chromosomes to the metaphase plate and designating the location of the future cytokinetic furrow. Thus as stated generally by Kant [9] and more specifically by Karsenti [10] "mitotic structures self-organize the dynamic properties required to act upon themselves to complete their teleological function...". For example, chromosomes organize the spindle for their own segregation, and the spindle midzone organizes the cytokinetic machinery to ultimately cleave itself in half during telophase. It is remarkable that predefined geographic cues are not needed to direct the spatial organization of events that define the metaphase plate or the cytokinetic furrow. Rather, it has been suggested that the dissipation of energy through the self-organizing properties of collective molecular deterministic interactions produces a spatial coordinate system that directs mitotic events [10,11].

The symmetry breaking required to successfully organize intracellular space for the equitable distribution of chromosomes and cytoplasm to daughter cells begins with the intrinsic asymmetry of the tubulin polymer with its plus and minus ends [12]. The polymerization of microtubules by the addition of tubulin subunits to the plus end and more slowly to the minus end, establishes the directional polarity that is utilized by plus (kinesin) and minus (dynein) directed motor proteins to bundle microtubules into asters, then bipolar structures during development of the mitotic spindle [10,13-15].

Proper assembly of a bipolar spindle, or accurate positioning of the cytokinetic furrow requires transmittal of spatial information across micron length scales within the cell. The drosophila embryo elegantly utilizes an intracellular diffusion gradient of Bicoid acting upon gap, pair rule, and segment polarity genes to organize discrete spatial patterns of development along the axis of the embryo [16]. During mitosis, intracellular gradients of phosphorylated stathmin [1], Ran-GTP [2], and most recently Aurora B kinase activity [3] act as spatial organizers by eliciting the discretely localized patterns of spindle, chromosome and cell membrane dynamics required for cell division [3,17,18]. The recent description of an interphase Pom1 kinase gradient in fission yeast adds to a growing list of intracellular gradients among eukaryotes, and indicates that intracellular activity gradients are a conserved regulatory paradigm [19].

Models of intracellular phosphorylation gradients have been proposed based on reaction-diffusion mechanisms, and dynamic changes in cell shape [20-22]. In the simplest model, (Figure 1a, b) a phosphorylated activator is generated from a local source and released into the cytoplasm where it diffuses away from the source until it encounters a phosphatase within the cytoplasm. The spatial separation of the source of the activator (kinase) from the inhibitor (phosphatase) produces a gradient of activity (phosphorylation) that is highest at the source [20,21].

**Figure 1:** **Theoretical intracellular phosphorylation gradients**. (A and B), a model proposed by Brown and Kholodenko [21,22] predicted that spatial separation of opposing activities (kinase and phosphatase (Ptase)) could produce a gradient (red to yellow) of activated substrates within the cell. The gradients could originate from the plasma membrane (A), or an intracellular structure such as chromatin (B), with the opposing activity homogenously distributed in the cytoplasm. The slope of the gradient is determined by α = √ k_p_/D where k_p _is phosphatase activity and D is the diffusion coefficient for proteins in the cytoplasm. (C), a model demonstrating how changes in cell shape can regulate intracellular gradients as proposed by Meyers and Odde [22]. Flattening of the cell at a protrusion or a trailing edge can cause localized increase in phosphorylation of a diffusible substrate, while an increase in cell thickness will cause dephosphorylation.

While most models of intracellular gradient formation follow similar assumptions, the situation in vivo is more complex [10]. Auto-activation, negative feedback and spatial regulation of the inhibitor contribute to the complexity of intracellular gradient formation. Moreover, the generation of intracellular mitotic gradients as spatial organizers in cultured cells or extracts that lack pre-localized cues illustrates the dynamic self-organization inherent to mitosis that interphase models of intracellular gradient formation do not address.

The concept of biological gradients has been most thoroughly studied during development when uncommitted cells are directed to adopt distinct patterns of differentiation in response to a morphogen. The notion that positional information could be translated into cell fate depending on the concentration of an organizing signal and the intrinsic responsiveness of the cell was first proposed by Wolpert [23]. In this model, cells closer to the origin of signal would be exposed to higher concentrations than those cells farther away. The graded concentration of morphogen induces unique developmental responses in target cells depending on their position in the gradient.

Before the biochemical identity of morphogens was known, attempts were made by investigators from a broad spectrum of disciplines to explain how patterns would emerge from the fertilized egg. Alan Turing's "Chemical Basis of Morphogenesis" [24] is a classic paper that established a conceptual and mathematic framework using simple chemical reactions to explain the genesis of patterns from a homogenous distribution of components. He postulated that minor instabilities such as stochastic fluctuations could be amplified to result in pattern formation if the new equilibrium were thermodynamically favored. To meet this requirement, he postulated a system of 2 morphogens in which morphogen X would need to be a catalyst for its own production. Its degradation would be proportional to the concentration of morphogen Y which would have a greater diffusion rate than morphogen X (Figure 2a, b). His diffusion reaction model predicted six distinct classes of "self-organizing patterns" including stationary or oscillating morphogen waves of various lengths [24]. At the time of the initial report in 1952 no biologic correlates were known, yet the model proposed by Turing would have a profound impact on the conceptualization of pattern formation during development. Turing's ideas would also have an impact on other physical and social sciences. More recently "Turing patterns" of sustained chemical non-equilibrium have been reproduced experimentally [25] and observed in nature [26]. Computer simulations of a Turing reaction-diffusion model were shown to predict the evolving pattern of stripes on the angelfish Pomacanthus as it grows [27,28], and to predict homogenous oscillations in the glycolytic pathway within cells [29].

**Figure 2:** **Models of pattern formation during development**. Alan Turing's model of pattern formation arising from the interaction of two morphogens is shown in (A). Red arrows indicate degradation, green arrow indicate autocatalysis. A key aspect of this model is that morphogens X and Y have different diffusion characteristics. (B), An example of a Turing pattern that was generated by a computer simulation of the model summarized in (A). Turing patterns in nature have been identified on squirrels, leopards, zebrafish and in the stripes of the marine angelfish pomacanthus, among others [27,28]. (C), The coloration of this scribbled rabbit fish resembles computer simulated Turing patterns as well as Turing patterns observed on other marine fish. (D), The Gier-Meinhardt model of pattern formation. Autoactivation is coupled to production of an inhibitor of longer range. As a result, a homogenous distribution of activator is unstable resulting in a gradient of activator.

The theory of self-organizing pattern formation as applied to biological development was significantly advanced by Gier and Meinhardt who expanded and refined Turing's reaction-diffusion concepts as applied to developmental biology. Inspired by the neurophysiology of lateral inhibition in visual processing inwhich local activation by a visual stimulus is coupled to production of an inhibitory effect that extends into surrounding areas, Mienhardt and Gier proposed that pattern formation could result from a self-enhancing activator of short range that produced its own inhibitor of longer range [30-32]. The activator/inhibitor reaction diffusion system proposed by Gier and Meinhardt predicts a self-regulating gradient of activator (Figure 2d). Moreover, an auto-catalytic activator coupled with a long range inhibitor has been shown not only to be sufficient, but absolutely required for pattern formation [32].

The morphogen concept was validated by studies of the drosophila syncitial embryo [16,33,34] in which maternal mRNA encoding the morphogen Bicoid is concentrated in the anterior pole of the syncitial cell. Intracellular diffusion of bicoid mRNA from anterior to posterior results in a gradient of translated Bicoid protein within the syncitial embryonic cell (Figure 3a, b). Bicoid protein is transcription factor capable of activating and inhibiting its target genes. Bicoid protein is also a translation factor capable of inhibiting translation of caudal proteins (*cad*) in the anterior region of the syncitial cell where Bicoid concentrations are highest [16,33]. Bicoid serves not only as an important conceptual model of morphogen induced patterning, but it is also the best characterized example of a diffusion mediated intracellular gradient [16,34]. In contrast, gradients within smaller cells (30 microns or less) cannot rely on diffusion alone but must also employ regulated zones of enzymatic activity for the addition or removal of post-translational marks [10,20,21].

**Figure 3:** **Intracellular gradients during Interphase**. (A), The drosophila syncitial embryo utilizes a gradient of bicoid mRNA (purple) that diffuses from the cephalad pole of the embryo, to the caudal pole. This results in a gradient of translated Bicoid protein (red) as shown in (B). (C), A gradient of Pom1 kinase is localized to the cell tips in *S. pombe*. As the cell grows, the gradient rescinds from the central region of the cell allowing activation of Cdr2 and downstream activation of Cdk-1 to trigger entry into mitosis (D) [38].

In nature, intracellular phosphorylation gradients are not confined to mitosis. Gradients of the dual specificity tyrosine kinase (DYRK) Pom1 have recently been described in fission yeast during interphase [35]. The intracellular gradient of Pom1 kinase reaches its maximum laterally at the cell tips where the highest concentration is anchored. The lowest point of the Pom1 gradient is in the mid-equatorial region - the future site of the cytokinetic furrow (Figure 3c). The Pom1 gradient maintains a relatively constant size throughout the cell cycle (approximately 8 um from the lateral cell tip). However, as *Pombe *cells grow and become more elongated, the gradient migrates laterally out of the central equatorial region, maintaining a constant gradient in the tip regions while reducing its concentration at the equator (Figure 3d). Pom1 kinase activity inhibits mid1, the *Pombe *equivalent of anillin - an actin binding protein that plays a key role in cytokinesis. Pom1 inhibition of mid1 persists until the cell has reached the proper size for mitosis and cytokinesis [36].

More recently, the Pom1 gradient has been shown to integrate control of cell size with regulation of the cell cycle. Pom1 inhibits Cdr2 in a concentration dependant manner [37]. Cdr2 through its inhibition of Wee1, promotes dephosphorylation of tyrosine 15 on CDK1 and mitotic entry. Pom1 acts to inhibit mitotic entry through this pathway when cells are small. As cells grow, the concentration of Pom1 in the equatorial midplane where Cdr2 is localized during interphase, begins to decrease. This relieves inhibition of Cdr2 resulting in reduced Wee1 activity, activation of CDK1 and entry into mitosis [37,38]. These experiments not only validate the existence of intracellular kinase activity gradients during interphase, but illustrate how intracellular gradients designate spatial information in order to coordinate independent events within the cell.

Spatial pattern generation during mitosis in the form of activity gradients occurs both before and after the metaphase to anaphase transition. The regulatory conditions that favor activity gradients during mitosis have received relatively little attention. With a focus on relationships that fit the reaction-diffusion paradigm of auto-activation coupled to long-range inhibition, the self-organizing properties of intracellular mitotic gradients are reviewed below. Known regulatory relationships will be re-examined to identify new potential interactions that might be predicted by established principals of pattern formation.

### Gradients Prior to Anaphase Onset

#### The OP18/Stathmin Phosphorylation Gradient

After simple intracellular phosphorylation gradients were shown to be theoretically possible if the kinase and opposing phosphatase were physically separated [20], Niethamer et al. described a phosphorylation mediated gradient of OP18/stathmin - tubulin interactions in mitotic HeLa cells utilizing a soluble Förester Resonance Energy Transfer (FRET) biosensor they named COPY (**C**FP - **OP**/stathmin - **Y**FP) [1]. Op18/stathmin is a unstructured 17 kilodalton cytoplasmic phospho-protein capable of binding 2 tubulin tetramers resulting in the sequestration of free tubulin (Figure 4a). A separate function of OP18/stathmin is to promote microtubule catastrophe [39]. Both of these properties of OP18/stathmin are inhibited by phosphorylation. OP18/stathmin is required for bipolar spindle assembly in *Xenopus *extracts however its role in mammalian cell mitosis is controversial [40].

**Figure 4:** **The OP18/stathmin phospho-gradient**. (A), The structure of alpha/beta tubulin subunits bound OP/18 stathmin. (B), Structure of the FRET sensor COPY. Cyan fluorescent protein (CFP) is bound to the N-terminus, and yellow fluorescent protein (YFP) is bound to the C-terminus of OP/18 stathmin. COPY adopts a rigid structure when bound to tubulin preventing FRET between CFP and YFP. Phosphorylation of COPY releases tubulin allowing interaction of CFP with YFP to produce FRET emissions. (C), A gradient of FRET emissions surrounding mitotic chromatin in HeLa cells is indicative of a gradient of phosphorylated OP/18 stathmin. (D), OP/18 stathmin could act as a local activator and long-range inhibitor of Aurora B kinase activation through effects on microtubule stability. Aurora B is activated by microtubules [43]. Phosphorylation of tubulin-bound OP18/stathmin increases free tubulin, inhibits its ability to induce microtubule catastrophe (promoting microtubule stability/polymerization), and increases OP18/stathmin diffusion by a factor of 2. Phosphorylated stathmin can then diffuse to the periphery where it is de-phosphorylated resulting in tubulin binding/sequestration and promotion of microtubule catastrophe. The gradient of Aurora B activity is shown in pink. (E), Computer generated Turing pattern based on the difference in diffusion coefficients of free and tubulin-bound OP18/stathmin [41].

COPY's designer's took advantage of OP18/stathmin's ability to assume a rigid elongated conformation when bound to tubulin [41], and attached fluorophores to either end (Figure 4B). Tubulin bound COPY adopts an elongated conformation and prevents CFP/YFP FRET. Phosphorylation of COPY causes release of bound tubulin and allows interaction of CFP with YFP to produce FRET emissions. Using COPY, Niethammer et. al. demonstrate a gradient of stathmin-tubulin interactions extending away from chromatin (Figure 4C) that is abolished when the phosphorylation sites on COPY are mutated from serine to alanine. This is the first demonstration of an intracellular gradient in mitosis mediated by protein phosphorylation. An important distinction between this phospho-gradient and the anaphase gradient discussed below is that a gradient of FRET activity was seen with biosensors attached to free, cytoplasmic OP18/stathmin, while a gradient was not seen with free cytoplasmic FRET reporters of anaphase Aurora B activity [3]. This discrepancy may relate to the different diffusion characteristics of the FRET biosensors. Fluorescence correlation spectroscopy analysis of stathmin-tubulin interactions has shown that OP18/stathmin's diffusion coefficient decreases by a factor of 2 when it is bound by tubulin [41]. In contrast, the untargeted cytoplasmc Aurora B FRET biosensor has no known molecular interactions that might affect its diffusion characteristics [3]. Thus, more limited diffusion of the substrate in concert with other factors such as spatial regulation of phosphatase activity, may allow visualization of an intracellular phospho-gradient with the soluble OP18/stathmin FRET biosensor.

More recently, chemical inhibition or depletion of Aurora B kinase was shown to prevent chromatin induced phosphorylation of OP18/Stathmin in *Xenopus *extracts [42], indicating that Aurora B kinase activity is required for the OP18/stathmin gradient during bipolar spindle assembly. How Aurora B kinase might contribute to a gradient of OP18/stathmin tubulin interaction is not clear. It is likely that additional factors including Aurora B activation as influenced by local interaction with kinetochore microtubules [43] may contribute to the regulation of OP18/Stathmin - tubulin interaction.

The stable gradient of OP18/Stathmin-tubulin interactions described by Niethammer extends over several microns. This is longer than would be expected if OP18/stathmin was in contact with centromere localized Aurora B or kinetochore localized PLK1. Indeed, FRAP analysis of GFP tagged Aurora B reveals rapid exchange between the centromeric and cytoplasmic pools of Aurora B [44]. This suggests that a gradient of activity in the soluble pool of Aurora B may contribute to the gradient of OP18/stathmin-tubulin interactions.

Given the recent demonstration that microtubules induce activation of Aurora B [43], it is possible to propose a reaction-diffusion model of the OP18/stathmin-tubulin gradient in which OP18/stathmin acts both as an activator and long-range inhibitor of Aurora B. Phosphorylation of OP18/stathmin in the proximity of Aurora B promotes stabilization of microtubules which in-turn activate Aurora B. Phosphorylation of OP18/stathmin by Aurora B releases it from tubulin subunits, allowing it to diffuse away from chromatin where de-phosphorylation and binding to tubulin subunits predominates. This would promote microtubule catastrophe and sequestration of tubulin subunits - limiting the concentration of microtubules available to activate Aurora B (Figure 4D). In this scenario, the increased diffusion of free OP18/stathmin vs. tubulin bound OP18/stathmin could establish a Turing style reaction-diffusion mechanism that promotes localized activation of Aurora B (Figure 4E). While other potential regulatory influences may contribute to a stable gradient of OP18/stathmin - tubulin interactions [45], Aurora B and OP18/stathmin-tubulin possess biochemical characteristics that could generate a self-organized gradient capable of promoting microtubule stability in proximity to chromatin, and microtubule catastrophe away from chromatin in order to guide bipolar spindle formation.

### The Ran Gradient

Microtubule nucleation and spindle assembly during mitosis are regulated by Ran-GTP [17,46]. While early reports suggested a link between Ran and formation of the mitotic spindle in yeast [47], more direct evidence came from the laboratory of Mary Dasso who demonstrated that RanBp1, a protein that facilitates the conversion of Ran-GTP to Ran-GDP, dramatically reduced microtubule growth in *Xenopus *extracts [48]. Ran mutants that inhibited RCC1 GEF activity (T24N) or that locked Ran-GTP in an active state by preventing GTP hydrolysis (G19V, L43E, Q69L) either prevented or promoted microtubule formation in extracts, respectively [46,48,49]. The effect of Ran on aster formation was initially shown to be indirect since Ran-GTP added to purified α and β tubulin did not promote microtubule formation [50]. Indeed, depletion of spindle assembly factors (SAF) like gamma tubulin and XMAP 215 prevents assembly of Ran induced asters in extracts [50]. This indicated that Ran's effects were mediated by cytoplasmic factors that promote microtubule polymerization and bundling. The breakthrough in understanding Ran's ability to promote aster formation and spindle assembly came when it was shown that Ran releases SAFs including TPX2 and other cargo from importin-β class nuclear transport receptors (NTR), also known as karyopherins [51]. There are nearly two-dozen identified regulators of mitotic spindle assembly that are bound by importin-β under the regulation of Ran-GTP [17,46]. In addition, Ran is capable of regulating the activity of the motor protein Eg5 directly [52], and the activity of Aurora A kinase indirectly through increasing TPX2 interaction with Aurora A. As described below, a gradient of Ran-GTP activity could provide the directional coordination of these activities around chromatin to promote generation of a functional bipolar spindle.

A gradient of Ran-GTP has been described surrounding chromatin in *Xenopus *extracts [4,7] and in mitotic human cells [2,17]. This results from the local production of Ran-GTP by RCC1 bound to chromatin. The local production and release of Ran-GTP by RCC1 results in a steep gradient of free Ran-GTP that is available to bind importin-β class NTRs causing release of SAFs in the immediate vicinity of chromatin (Figure 5). This catalyzes nucleation of microtubules adjacent to chromatin, and results in the longer-range stabilization of microtubules distal to chromatin [7]. Because RCC1 itself is a cargo of importin-β, the increase in Ran-GTP on the surface of chromatin promotes additional delivery of RCC1 to chromatin in a positive feedback loop. The positive feedback regulating RCC1 localization to chromatin is one of several hallmark features of RCC1 regulation that are characteristic of self-organizing regulators that must break the symmetry of their local environment to create spatial patterns [10,24,32].

**Figure 5:** **Ran-GTP gradient**. Local production of Ran-GTP by chromatin bound RCC1 produces a series of subordinate Ran-GTP dependent gradients that organize development of the mitotic spindle around chromatin. (A), Localized Ran-GTP production by RCC1 releases spindle assembly factors (SAF) from Importin beta around chromatin where they nucleate microtubules. (B), Diagram of Ran-GTP, SAF, Ran-GTP-Importin beta, and Ran-GTP-Importin beta-RanBP1 diffusion gradients that convey positional information to components of the developing mitotic spindle.

The spatial geometry of the mitotic Ran-GTP gradient has been visualized by a variety of Ran sensitive FRET biosensors in *Xenopus *extracts [7] and intact cells [2]. Utilizing a Ran binding domain peptide and a importin-β binding domain peptide, Kalab, Wiess and Heald developed biosensors that emit low FRET signal (Ran binding peptide) or high FRET signal (importin-β binding peptide) when bound by Ran-GTP (Table 1). They observed a gradient of FRET signal centered on chromatin measuring approximately 10 - 12 microns in *Xenopus *extracts that was attributed to a localized gradient of Ran-GTP generated by chromatin bound RCC1 [4]. Caudron et. al. showed that a gradient of Ran could generate differential responses that were concentration dependant over a long range. They demonstrated that the concentration threshold for microtubule nucleation is distinct from that for microtubule stabilization in *Xenopus *extracts. This was accompanied by the demonstration of a long-range gradient of Ran-GTP-importin-β interaction as visualized by fluorescence lifetime imaging (FLIM) of alexa 488 labeled Ran and CFP labeled importin-β. The distinct concentration dependant responses of microtubule nucleation and microtubule stabilization were correlated with the gradient of Ran-GTP-importin-β to illustrate that graded concentrations of Ran-GTP and its binding partners provided spatial coordination of microtubule regulators during spindle assembly [7]. The long-range gradient of Ran-GTP-importin-β interaction also provides a mechanistic explanation for the known long-range interactions between chromatin and centrosome nucleated microtubules observed in *Xenopus *extracts [53].

**Table 1:** FRET reporters used to study intracellular mitotic gradients

Name	Probe for:	Structure	Reference
YRC	Binding/release of Ran	YFP-***Ran Binding Domain***-CFP	Kalab [4]

YIC	Binding/release of Importin Beta cargo	YFP-***Importin-β Binding Domain***-CFP	Kalab [4]

COPY	Tubulin binding to Stathmin	CFP-***OP18/Stathmin***-YFP	Niethammer [1]

Alexa488-Ran	Ran/Importin Beta interaction	***Ran***-Alexa 488	Caudron [7]

Cy3-Importin-*β*	Ran/Importin Beta interaction	***Importin-β***-Cy3	Caudron [7]

RANGO	Binding/release of Importin Beta cargo	EYFP- ***Importin-β Binding Domain***-Ceru.	Kalab [2]

ABAR	Aurora B activity	***Targeting***-CFP- ***FHA2-Substrate***-YFP	Lampson et. al [3]

ABAR, Aurora B activity reporter; Ceru., cerulean; CFP, cyan fluorescent protein; EYFP, enhanced yellow fluorescent protein; RANGO, Ran-regulated Importin beta cargo; YFP, yellow fluorescent protein; YIC, YFP-Importin-Beta Binding Domain-CFP; YRC, YFP-Ran Binding Domain-CFP.

The presence of the Ran-GTP gradient in HeLa cells was confirmed by Kalab et al. Utilizing FLIM, and a FRET biosensor built around the importin-β binding domain (Table 1), they demonstrated a higher Ran-GTP concentration and lower importin-β cargo binding around mitotic chromatin in HeLa cells [2]. Comparison of the dimensions of the gradient in HeLa cells (3-4 microns) to that observed in *Xenopus *extracts (10 - 12 microns) reveals a remarkable difference. However, in both cases the gradient of free importin-β cargo extended to the spindle poles, demonstrating the remarkable robustness of the Ran-GTP gradient across different species [2,4,17]. In HeLa cells, FLIM is able to detect a relatively small but significant gradient (13% increase) of Ran-GTP around mitotic chromatin. Increases in Ran-GTP of this magnitude are sufficient to nucleate microtubules in *Xenopus *extracts, even in the presence of free importin-β cargo [2,17].

**RCC1**, the only known Ran GEF, forms 7 characteristic β-propeller structures (individually referred to as RCC1 like domains, RLDs). The structure of RCC1, with its 7 β-propeller domains, resembles a French crueler doughnut [54]. RCC1 has unstructured amino and carboxy terminal tails. Localization of RCC1 to chromatin is highly dynamic with rapid exchange of chromatin bound and unbound forms [55]. RCC1 binding to chromatin is mediated by its amino terminal tail, and through interaction of its RLDs with the core histone domains of H2a and H2b [56]. Ran binding to RCC1 occurs on the distal face of the doughnut relative to chromatin, and histone binding occurs on the proximal face, from which the amino and carboxy tails protrude (Figures 5A, 6A).

**Figure 6:** **Localization-catalysis coupling of RCC1 self-organizes the Ran-GTP gradient around chromatin**. (A), Binding of substrate (Ran-GDP) to RCC1 causes a conformational change in the N-terminal tail of RCC1 to promote binding of RCC1 to chromatin [60]. Exchange of GDP for GTP promotes release of Ran and RCC1 from chromatin. (B), Ran flux at the kinetochore could promote tight association of RCC1 and the RSSU complex to the outer centromere/kinetochore region with reciprocal self-reinforcement. Localized Ran-GTP production promotes RSSU binding to the kinetochore, and local production of Ran-GDP by RSSU promotes tight association of RCC1 to chromatin.

The amino terminal tail of RCC1 has several unique features that regulate the localization of RCC1 to chromatin. It contains a bipartite NLS that binds importin-α, an adapter protein that facilitates binding to importin-β. Phosphorylation of the NLS by CDK1 results in release of RCC1 from the importin-β complex so it can bind to chromatin [57]. mRNA splice variants of RCC1 result in 4 different isoforms that differ in their NLS, affinity for importin-β and ability to be phosphorylated by CDK1 [58]. In addition, amino terminal proline/serine methylation increases RCC1 binding to DNA [59]. While it had been shown that binding of RCC1 to chromatin increases its catalytic activity [55], and that RCC1 bound to the apo (nucleotide-free) form of Ran increases its affinity for chromatin [55], the mechanistic basis for this relationship remained poorly understood until recently. Taking advantage of the unstructured carboxy and amino tails of RCC1 that co-occupy its proximal face, Hao and Macara attached CFP and YFP to them to create a FRET biosensor sensitive to changes in the mobility of the amino terminal tail. They not only show that RCC1 binding to DNA is dependant on the amino terminal tail and its methylation, but that RCC1 binding to histones is inhibited by the amino tail, unless RCC1 was bound by Ran-GDP. Furthermore, binding of Ran-GDP to the RCC1 FRET biosensor inhibited FRET - indicating that Ran binding produces a conformational change in the amino tail that promotes RCC1 binding to chromatin. Ran-GDP had no effect on histone binding when RCC1 lacked the amino tail [60]. Together, these observations demonstrate that RCC1 binding to chromatin is facilitated by a conformational change in its amino terminal tail that occurs upon Ran-GDP binding. Release of newly activated Ran-GTP restores the basal conformation of the tail and promotes release of RCC1 from chromatin by reducing RCC1 affinity for histones (Figure 6a). These results are consistent with earlier data demonstrating that production of the Ran-GDP-RCC1 ternary complex is coupled to chromatin binding [55]. This mechanism of Ran-GDP dependant targeting of RCC1 illustrates how catalytic production of an activator can reinforce the geographic localization of a gradient's origin, underscoring the self-organizing nature of intracellular mitotic gradients as engines of positional information.

Ran-GTP flux, i.e. the progression of Ran through the full cycle of guanine nucleotide binding states, may contribute to RCC1 regulation at the kinetochore [46]. Crm1, also known as exportin1, is a karypherin of the importin family who's interphase function is to shuttle proteins containing a nuclear export sequence out of the nucleus in a Ran-GTP dependant manner [61]. During mitosis, Crm1 binds a complex containing RanBP2, RanGap1 and Sumo (RRSU) that is targeted to the kinetochore by Ran-GTP [62]. The precise function of RanGap1 at the kinetochore is still unclear. However, 'flux' of Ran-GTP at the kinetochore could have several local consequences including: increased local Ran-GTP production; tighter association of RCC1 with chromatin; and a localized increased release of SAF's at the kinetochore. Increased Ran-GTP production may also stabilize RRSU localization, resulting in a self-reinforcing regulatory circuit in which flux enhances RRSU binding at the kinetochore (Figure 6B). Although diffusion might reduce the long-range consequences of Ran-GTP flux at kinetochores, it is likely that flux plays a role in regulation of microtubule kinetochore attachments since the loss of RanGap1 from the kinetochore results in severely abnormal attachments demonstrating extreme merotely [62]. Alternatively, Crm1, RanGap1, or other members of the RSSU complex may have additional roles in kinetochore function. Although little is known about the binding of RCC1 to the specialized chromatin that characterizes the centromere, the localization of RSSU complex containing RanGap1 to the centromere suggests that Ran-GTP flux could facilitate this interaction. Additional biochemical studies and mathematical modeling are needed to evaluate the potential significance of Ran-GTP flux at the kinetochore.

The emerging concept is that generation of Ran-GTP by chromatin bound RCC1 establishes a series of concentric subordinate gradients that consist of Ran-GTP, liberated spindle assembly factors, Ran-importin-β, and Ran-importin-β-RanBP1. These complexes exert position specific influence on microtubule regulation to focus bipolar spindle formation around mitotic chromatin. Ran-GTP production is catalytically coupled to RCC1 localization, ensuring that the biochemical origin of the gradient is targeted to mitotic chromatin. Additionally, Ran-GTP mediated targeting of regulatory complexes (Crm1, RSSU) to specific sites such as the centrosome and kinetochore, indicates that Ran regulation is more complex than can be explained by a generalized gradient alone. Existing data support two overlapping modes of Ran spatial regulation for spindle assembly - one that is gradient mediated, and one that is Ran GTP targeted.

In order for the Ran-GTP gradient to function as robustly as demonstrated experimentally, some form of regulatory inhibition appears to be required. This would insure that the correct levels of Ran are produced to maintain spatial integrity of the Ran-GTP gradient - whether it forms in *Xenopus *extracts, or somatic human cells. Currently no feedback inhibition in the generation of the Ran-GTP gradient has been demonstrated. It will be important to determine if the Crm1-RanBP2-RanGap1 complex could contribute to gradient stability and/or robustness by providing negative feedback, or through Ran-GTP flux.

### Gradients After Anaphase Onset

#### The Anaphase Aurora B Phosphorylation Gradient

Maintenance of genome integrity during cell division requires coordination of chromosome segregation and cytokinesis, so that the daughter cells inherit exactly one copy of each replicated chromosome. Anaphase, which has been called the beginning of cytokinesis, is a complex regulatory period that heralds the end of mitosis [63-65]. Degradation of cyclin B and securin initiate a cascade of anaphase events that include separation of sister chromatids [66-68], activation of cellular phosphatases [69], reorganization of the mitotic spindle [70,71], segregation of chromosomes toward the poles [72,73] development of the spindle midzone [74], and accumulation of active RhoA at the site of the future cytokinetic furrow [75].

Anaphase also triggers departure of the Chromosome Passenger Complex (CPC) from the inner centromere. It next localizes to its final destination - the parallel-opposed microtubules of the spindle midzone (Figure 7) [76]. The anti-parallel microtubules located between segregating chromatids in the spindle midzone are stabilized by microtubule associated proteins (MAPs) and bundled by motors proteins to form the core of the anaphase spindle midzone. Pole-ward force exerted on anti-parallel midzone microtubules by motor proteins lengthens the spindle, further separating the spindle poles and their attached complement of chromosomes during anaphase B [77]. The spindle midzone, which also serves to concentrate key regulators of cytokinesis (PRC1, centralspindlin, CPC, PLK1), produces a signal that directs ingression of the cytokinetic furrow [3,74,78-83]. Thus the spindle midzone, a self-organized structure in its own right, coordinates chromosome segregation and cytokinesis.

**Figure 7:** **Chromosome passenger complex (CPC)**. (A), Localization of the CPC during mitosis in *Xenopus *XTC cells: green, tubulin; blue, Dapi; red, Aurora B. Arrow points to midzone localization of Aurora B (reproduced with permission from Bolton et al, [129] ASCB). (B), Model of the CPC depicting the relationship of survivin and borealin to INCENP's N-terminal region. The C-terminus of INCENP contains the "IN Box" that tightly binds Aurora B. (C), Model of the two-step activation of CPC Aurora B kinase activity. Initial phosphorylation of the T-loop on Aurora B results in partial activation. Phosphorylation of INCENP at Serine 850 results in full activation. Structural and biochemical studies suggest that Aurora B is trans-autoactivated (c-terminus of INCENP shown in blue). (D), Aurora B phosphorylation target motifs.

How does the spindle midzone direct the initiation and progression of the cytokinetic furrow at the cell cortex more than 5 - 20 microns away? Immuno-fluorescent and FRET imaging data demonstrate a gradient of Aurora B kinase activity originating from the spindle midzone. Increasing evidence suggests this gradient acts as a spatial organizer that designates the location of the cytokinetic furrow while regulating anaphase spindle and chromosome dynamics [3,18,71].

Aurora B is a serine/threonine kinase that is conserved in all eukaryotes. It is required for proper kinetochore attachment, kinetochore bi-orientation and chromosome segregation. During anaphase, Aurora B kinase activity is required for proper spindle midzone structure and composition, as well as successful completion of cytokinesis [82-89]. Aurora B combines with INCENP, survivin and borealin to form the "chromosome passenger complex". The chromosomal passenger complex was so named because of its unique temporal localization pattern during mitosis [76]. The CPC forms in the nucleus in G2 and localizes along the length of condensing chromosomes in prophase. It then concentrates at the inner centromere during prometaphase and metaphase. The CPC disembarks from the inner centromere shortly after anaphase onset and localizes to midzone microtubules. In metazoans this precedes the appearance of Aurora B at the inner surface of the equatorial cell membrane where the cytokinetic furrow will later form [84,90]. The CPC ultimately becomes concentrated in the telophase midbody where it plays a role in cell abscission [89,91]. The proteins that compose the CPC facilitate regulation of Aurora B kinase through the stimulation of kinase activity (INCENP and survivin) or targeting Aurora B to specific substrates (INCENP, survivin and borealin) [92,93]. The CPC has an essential role in cytokinesis. Depletion of any member of the complex will cause a cytokinetic defect [94-97].

Aurora B binds INCENP to form the catalytic core of the CPC. Existing data suggest a two-step process of Aurora B kinase activation. Binding to the "IN box" on INCENP's carboxy terminus is required for activation of Aurora B above a minimal level. This is associated with phosphorylation of threonine 232 in the activation domain of Aurora B. Subsequent phosphorylation of INCENP at serine 850 (*Xenopus*, serine 893 and 894 of human INCENP) is required for full activation of Aurora B [98,99]. Serine 850 is surrounded by a well-characterized Aurora kinase phosphorylation motif (Figure 7D). Based on the crystal structure of Aurora B bound to INCENP, phosphorylation of INCENP on S850 by Aurora B is predicted to occur via trans-auto-activation [99].

Within 60 seconds after anaphase onset, the Aurora B complex relocates from the centromere to microtubules in the spindle midzone [84]. Transfer of the Aurora B complex to the spindle midzone requires destruction of Cyclin B [84]. MKLP-2, a class 6 kinesin that shows limited homology with MKLP-1, acts as a docking receptor for the Aurora B complex on midzone microtubules. RNAi depletion of MKLP-2 prevents Aurora B complex binding to the spindle midzone and blocks cytokinesis [3,100]. Although the Aurora B complex is an integral part of the spindle midzone and essential for cytokinesis, almost nothing was known about the regulation of its activity during anaphase until recently.

#### Evidence for an Aurora B phosphorylation gradient in anaphase cells

Initial insights regarding anaphase Aurora B activation were provided by analysis of the spatial pattern of phosphorylation of Aurora B substrates during anaphase. A gradient of Aurora B activity was suggested when radiation induced anaphase lagging chromosomes in HeLa cells retained 2.5 - 10 fold higher phosphorylation of histone H3 at serine 10 (H3(S10)) compared to chromatin that had segregated to the poles (Figure 8). A similar gradient pattern of H3(S10) phosphorylation was observed in non-treated HeLa cells (Figure 8), as well as other human and *Xenopus *cell lines [3]. The H3(S10) phosphorylation gradient was also observed in Drosophila syncitial embryos, however, that gradient is lost from anaphase after cellularization [101]. Data from a range of organisms and cell lines now indicate that the anaphase H3(S10) phosphorylation gradient represents a universal feature of mitosis in higher eukaryotes [3,101-104]. The anaphase gradient pattern of phosphorylation has been observed on other Aurora B substrates including MCAK at serine 196 [105], and is remarkable because it does not appear to be confined to substrates contacting midzone microtubules where Aurora B is concentrated. Rather the phosphorylation pattern appears to reflect a soluble gradient of Aurora B kinase activity.

**Figure 8:** **A gradient of H3 (S10) phosphorylation is evident during anaphase in radiated (A, B), and non-radiated HeLa cells (C)**. HeLa cells were treated with 8 Gray and fixed for immunofluorescence 16 hours later. Note that DNA damage does not appear to prevent Aurora B kinase activity during the first mitosis following radiation. Lagging chromosomes reveal a positional gradient of H3(S10) phosphorylation that is also evident on untreated HeLa cells. The arrow in the third panel in B indicates loss of Aurora B staining in the central-most region of the spindle midzone. Line graphs in (B) and (C) are intensity profiles through the plane indicated by the green line in figures (B) and (C). Note the peak of H3(S10) phosphorylation intensity is closer to the spindle midzone than the peak of Dapi intensity.

To better characterize the anaphase dynamics of Aurora B kinase activity, an Aurora B Activity Reporter (ABAR) was developed by Mike Lampson and Tarun Kapoor [3] based on the FRET biosensor designed to report PKC activity [106]. The carboxy-terminus of ABAR consists of an Aurora B phosphorylation consensus sequence flanked by an FHA2 domain immediately upstream, and YFP in the extreme C-terminus. The amino terminus of ABAR contains a intracellular localization targeting domain and CFP (see Table 1). Phosphorylation of ABAR by Aurora B prevents interaction of CFP and YFP and therefore prevents FRET. De-phosphorylation of ABAR or inhibition Aurora B activity promotes FRET. Cells expressing ABAR targeted to chromosome arms or centromeres demonstrated a gradient of FRET signal during anaphase (Figure 9). No FRET gradient was observed with freely diffusible, cytoplasmic, non-targeted ABAR. This latter finding is consistent with models of intracellular phosphorylation gradients by Kholodenko et al. that predict protein diffusion would have a negative effect on gradient stability [20,21]. In this instance, rapid intracellular diffusion of both kinase and substrate may prevent detection of a gradient.

**Figure 9:** **FRET reporters reveal a positional gradient of phosphorylation during anaphase**. Phosphorylation of the Aurora B activity reporter ABAR inhibits FRET emissions. (A), centromere targeted ABAR FRET probe; (B,) chromatin targeted ABAR FRET probe; (C), cytosolic, untargeted ABAR FRET probe; (D), Chromosome targeted PLK1 activity FRET probe indicating no evidence of a gradient of PLK1 kinase activity.

Inhibition of Mad2 in ABAR expressing HeLa cells generated lagging chromosomes, and increased the positional distribution of ABAR across the anaphase spindle. This allowed separation of the influences that time in anaphase, or chromosome position along the spindle, might have on FRET signal intensity. This analysis revealed that phosphorylation of ABAR was primarily a function of position along the spindle (i.e. distance from the midzone) rather than time in anaphase, consistent with a spatial gradient of kinase activity [3].

Unlike the intracellular gradient models that are dependant on cell geometry as proposed by Odde et. al [23], the Aurora B activity gradient persists even during anaphase in monopolar cells. In monopolar cells produced by sequential inhibition of Eg5 and CDK1, there is no spindle midzone yet Aurora B accumulates on ectopic microtubules that resemble the periphery of an aster [107,108]. This is accompanied by a directional gradient of H3(S10) phosphorylation on chromatin, and followed by ingression of a cytokinetic furrow at the gradient maximum, located opposite of chromatin moving toward the pole [3].

Together, these observations demonstrate that a gradient of Aurora B kinase activity can be observed on endogenous and exogenous Aurora B targets in a variety of cell types, and it appears to play a central role directing the location of the cytokinetic furrow. Anaphase mis-localization of Aurora B prevents gradient formation [3]. Thus the gradient depends on the subcellular localization of Aurora B kinase and its substrates such that phosphorylation of a substrate reflects its position relative to the spindle midzone. Experiments in monopolar cells demonstrate that the gradient is independent of spindle bipolarity, but nevertheless spatially coordinates the dynamic relationship between furrow ingression and poleward movement of anaphase chromatin [3,107,108].

Experiments utilizing Hesperadin, a selective Aurora kinase inhibitor, provide several insights into the anaphase regulation of Aurora B and the resulting anaphase phosphorylation gradient. Brief (8 minute) exposure to Hesperadin reduces H3(S10) phosphorylation in anaphase cells - confirming FRET evidence for opposing Aurora B kinase and phosphatase activities during anaphase. This is in contrast to prometaphase, where longer incubations in Hesperadin are needed to reduce H3(S10) phosphorylation [3] due to CDK1 induced phosphatase inhibition [69]. The reduced level of H3(S10) phosphorylation following brief exposure to Hesperadin during anaphase is associated with loss of the gradient pattern of H3(S10) phosphorylation in 100% of anaphase cells. This indicates that spatial regulation of phosphatase activity *alone *cannot account for the phosphorylation gradient observed on native substrates, and suggests that a gradient of Aurora B *activity *is required. Finally, Hesperadin treatment perturbs Aurora B localization and midzone microtubule structure. Midzone microtubules are fewer and/or more disorganized, and Aurora B coalesces into large patches that extend beyond the midzone (Figure 10c). Thus, Aurora B kinase activity during anaphase appears not only responsible for the observed phosphorylation gradient, but is also required to maintain spindle midzone structure and its own localization [94,96].

**Figure 10:** **Microtubule dependant autoactivation in the spindle midzone generates a gradient of Aurora B activity**. (A), control; (B), brief exposure of HeLa cells to Nocodazole causes loss of midzone microtubules, displacement of Aurora B from the midzone, and loss of the histone H3 (S10) phosphorylation gradient. Similarly, inhibition of Aurora B activity by treatment with Hesperadin in (C) results in displacement of Aurora B (arrow), loss of midzone microtubule organization, and loss of the histone H3 (S10) phosphorylation gradient. (D - F), microtubules and Aurora B kinase activity are required for full activation of Aurora B in the spindle midzone. Brief exposure of *Xenopus *S3 cells to Nocodazole (E), or Hesperadin (F) results in disruption of midzone microtubules and loss of INCENP S850 phosphorylation; (D), control. (G), Aurora B and midzone microtubules physically interact. Proximity-ligation assay (P-Lisa) was used to detect physical interaction between Aurora B and microtubules in anaphase *Xenopus *S3 cells. Tubulin is stained green, the kinetochore marker Ndc80 is stained blue and P-Lisa product, demonstrating contact between Aurora B and microtubules in the midzone, is shown in red (C, G reproduced with permission from Fuller et al, [3] NPG).

#### Auto-activation and positive feedback characterize anaphase Aurora B activation

Aurora B activation during anaphase was initially suggested by Goto et.al. who demonstrated midzone localization of antibodies to INCENP phospho-serine 894-895, an indicator of Aurora B kinase activation [109]. More recently, phospho-antibodies to INCENP S850 (the equivalent site in *Xenopus*), were used to study anaphase activation of Aurora B in *Xenopus *S3 cells. Brief exposure to Hesperadin abolished the normally robust pattern of INCENP S850 staining in anaphase cells (Figure 10f). This demonstrated that S850 phosphorylation itself is dependant on Aurora B kinase and opposing phosphatase activities, and that full activation of Aurora B kinase, through phosphorylation of S850, occurs during anaphase. Thus Aurora B appears to be auto-activated in-trans in the anaphase spindle midzone. Aurora B's ability to trans-activate can be also be demonstrated in vitro by the addition of bivalent anti-INCNEP antibodies to preparations of INCNEP and Aurora B. Aurora B activation is catalyzed by clustering of Aurora B/INCENP complexes, but it does not occur following addition of univalent antibody [110].

Aurora B activation during anaphase is localized to midzone microtubules (Figure 10) [3,109]. The nocodazole induced loss of H3S10 phosphorylation from anaphase chromatin suggests that anaphase activation of Aurora B kinase is dependant on midzone microtubules. Indeed, nocodazole treatment of *Xenopus *S3 cells reduces anaphase INCENP S850 phosphorylation by 85% [3]. This is consistent with the known ability of microtubules to activate Aurora B in vitro [43]. Direct interaction of Aurora B kinase with anaphase midzone microtubules can be detected by proximity ligation in situ assay (P-Lisa) [111]. Anaphase P-Lisa signal co-localizes with INCENP S850 and Aurora B T232 phosphorylation - both markers of Aurora B activation [3,98,99,112]. Together these data argue that the spindle midzone functions as a structure based auto-feedback loop for Aurora B activation. Aurora B activation stabilizes midzone microtubules, and midzone microtubules catalyze Aurora B activation. This occurs in concert with trans auto-activation of the CPC by phosphorylation of Aurora B at T232 and INCENP at S850. This positive feedback loop at the origin of the gradient is precisely the type that would have been predicted by the self-organizing pattern formation concepts originally proposed by Turing [24] and further developed by Gier and Meinhardt [29,31,32]. The concept that self-organizing systems use phosphorylation gradients to establish positional information for intracellular events is an important new principle that has wide ranging biological implications.

Existing data support a model in which the kinesin MKLP-2 could carry the Aurora B complex to the central midzone region where the kinase could be activated and released to generate a gradient of soluble kinase activity (Figure 11). Other kinases including AKT are released following activation at the cell membrane [113]. Rapid inactivation of released Aurora B by soluble phosphatases and/or degradation would generate a gradient, although spatial inactivation of Aurora B has not yet been demonstrated. Alternatively, because Aurora B can auto-activate in trans, the gradient of activity could simply reflect the concentration of Aurora B as it is carried down microtubules from two directions.

**Figure 11:** **Alternative models of anaphase Aurora B kinase activation and gradient formation**. Diagrams A and B depict models of the anaphase midzone. During anaphase, MKLP2 binds the chromosome passenger complex (CPC) to midzone microtubules. MKLP2 plus-end directed motor activity concentrates the CPC in the central most region of the spindle midzone resulting in Aurora B activation such that peak activity is achieved in the center of the spindle midzone. Contact with midzone microtubules, co-activators such as TD60, and/or trans-autoactivation might contribute to Aurora B activation. (A), upon full activation of Aurora B kinase, the CPC is released either through loss of MKLP2-microtubule interactions, or de-polymerization/severing of central midzone microtubules resulting in dissociation of CPC-MKLP2 complexes. This latter model might explain the curious absence of microtubule-bound Aurora B in the central most region of the spindle midzone (Figure 8b). CPC with fully activated Aurora B kinase then diffuses away from the midzone to activate Aurora B in the soluble pool, encounter inactivating phosphatase activity, or be degraded. Alternatively, as in (B), the soluble cytoplasmic pool of CPC diffuses toward the spindle midzone where it is trans-activated by midzone bound CPC with highly active Aurora B. Cellular phosphatase activity (not shown for simplicity) should play a major role in regulation of the Aurora B activity gradient (see text for additional details).

Existing data do not address the long-range inhibition of Aurora B needed to produce the stable gradient of declining phosphorylation that is observed. Because phosphatase activity affects so many aspects of anaphase progression, simple chemical or genetic phosphatase inhibition may be insufficient to identify the phosphatase or its regulatory partners that contribute to the gradient of Aurora B activity. PP1 and PP2a have been isolated in complexes containing Aurora B [114,115], and Aurora B itself contains at least two PP1 interaction motifs [116]. Additional work is needed to determine whether there is a spatial dimension to phosphatase activity, and if so what regulatory conditions are required, and how they might contribute to the establishment or maintenance of a phosphorylation gradient.

#### Potential roles of the gradient in anaphase

All of the conditions that disrupt the anaphase H3(S10) phosphorylation gradient also block cytokinesis [3,85,93,117-120]. Under certain experimental conditions, there are two independent signals that establish the cytokinetic furrow: one from astral microtubules and another from the spindle midzone [79]. Both signals depend on Aurora B. After physically blocking the midzone from the cell cortex, Wang and colleagues demonstrated that astral microtubules can deposit Aurora B to the central region of the cortex [84]. Conversely, low dose nocodazole treatment resulting in selective loss of astral microtubules had no effect on initiation or progression of cytokinesis (William Bement, personal communication). How the spindle midzone, in the center of the cell, can signal to the cortex over micron length-scales has remained a mystery. The generation of a soluble gradient of Aurora B activity is one potential mechanism for communicating over the large distances required to specify furrow location.

Experimental displacement of the spindle midzone from the equator, or juxtaposition of asters from two separate spindles in dikaryons or heterokaryon fusions, results in formation of a functional ectopic cytokinetic furrow [121-124]. Similarly, repositioning a patch of non-equatorial cell membrane close to midzone microtubules produces localized RhoA activation and ectopic furrow formation in the repositioned membrane [75]. These results suggest that specification and progression of the cytokinetic furrow is not regulated by a pre-localized complex, but by a self-organizing system. A central component of many developmental self-organizing systems are auto-activation and auto-inhibitory loops that produce stable gradients of an activator/organizer. The auto-activation and stable gradient formation that characterize anaphase regulation of Aurora B kinase activity recapitulate core regulatory elements of self-organizing systems [32]. This property, taken together with demonstrations of the self-organizing nature of the signal directing cytokinesis and its dependence on Aurora B activity, support the notion that the gradient of Aurora B activity might be the midzone signal responsible for directing the position of the cytokinetic furrow.

## Conclusion

Mitotic gradients are directional fields of intracellular activity that designate regions of the cytoplasm for localized progression of specific mitotic events. They are not dependant on pre-existing positional marks within the cell or plasma membrane. Rather, they utilize auto-activation and most likely auto-inhibition to generate fields that establish positional information. The mitotic gradients described thus far are centered on mitotic structures such as chromosomes or the spindle midzone. As yet there are no proven examples of pure freestanding Turing type chemical disequilibriums during mitosis. However, applying general principals of pattern formation to the analysis of mitotic gradients identifies common regulatory themes based on the biochemical interactions rather than the properties of a single molecule.

This review has highlighted several similarities between the RCC1-Ran system and the CPC. Both are associated with chromatin. Both utilize self-enhanced localization at the origin of their respective gradients, and both systems regulate the sorting of macromolecular complexes into teleologically significant, and geographically distinct regions of the cytoplasm. While the RCC1-Ran-RanGap1 system utilizes karyopherins to spatially organize the cytoplasm both during interphase and mitosis, Aurora B accomplishes spatial organization prior to anaphase by regulating kinetochore-microtubule attachments and spindle dynamics to regulate "positioning" of chromosomes at the metaphase plate [46,48,76]. After anaphase onset, Aurora B activity regulates RhoA localization to position the cytokinetic furrow [108,125,126].

An immediate challenge is to identify additional core components of these self-organizing circuits in molecular terms. In particular, to determine if the activator-induced inhibition, as theoretically predicted to support robust gradient formation, can be identified. For both RCC1-Ran and the CPC, spatial regulation of an inhibitory activity seems likely. Additional work is needed to demonstrate whether Ran-GTP production also increases RanGap1 activity to generate a long-range inhibitory signal. A similar caveat exists for the phosphorylation gradients produced by the CPC. Phosphatase activity, specifically that of PP1 and PP2a, has been shown to oppose Aurora B kinase in genetic and biochemical systems [114,115,127-129]. Experiments to elucidate the spatial regulation of CPC activity by phosphatases are in progress [127].

Intracellular gradients appear to coordinate distinct events and pathways within the cell. Whether it's coordinating cell size and cell cycle progression during G2 in *Pombe*, or chromosome movement and cytokinesis during anaphase in vertebrate cells, gradients of activity prevent catastrophic dis-coordinate progression of key events in order to ensure proper execution of cell division. Hence, gradients may represent a novel tumor suppressor mechanism as well as a potential therapeutic target for cancer treatment.

## Competing interests

The author declares that he has no competing interests.

## Authors' contributions

BGF wrote the manuscript and produced all of the figures except where portions were reproduced with permission (figures 7 and 10)
